The article "The Relationship between Body Composition and Bone Mineral Density of Female Workers in A Unit of Tai'an" was retracted in 2023. Reasons: signs of a paper mill; suspected computer-generated content; unreliable results or conclusions; concerns about the data.

# The Relationship between Body Composition and Bone Mineral Density of Female Workers in A Unit of Tai'an

**DOI:** 10.1155/2022/1011768

**Published:** 2022-02-08

**Authors:** Yan Wang, Siqi Wang, Zhengxiu Chen, Zhangshen Ran

**Affiliations:** ^1^Department of Endocrinology, The Second Affiliated Hospital of Shandong First Medical University, Ta'ian, 271000 Shandong, China; ^2^Regular Physical Examination Centre, The Second Affiliated Hospital of Shandong First Medical University, Tai'an, 271000 Shandong, China

## Abstract

**Objective:**

To explore the relationship between body composition and bone mineral density (BMD) of female workers in a university of Tai'an.

**Methods:**

This study randomly selected 90 female employees in a university of Tai'an. The body composition was monitored by body composition analyzer (inbody770), and the lumbar bone mineral density was monitored by dual energy X-ray absorptiometry (BMD model). The data were analyzed by SPSS 22.0 statistical software.

**Results:**

With the increasing of body mass index (BMI), BMD of female lumbar spines 1-4 (L1-4) increased gradually. Spearman correlation analysis showed that BMI, skeletal muscle mass, upper limb muscle mass, trunk muscle mass, lower limb muscle mass, and whole-body phase angle were positively correlated with L1-4BMD. Age was negatively correlated with L1-4BMD. Linear regression analysis showed that age was a negative factor of L1-4BMD, and skeletal muscle mass was a protective factor of abnormal bone mass, especially lower limb muscle mass.

**Conclusions:**

Lower limb muscle mass is a protective factor of female BMD. Strengthening physical exercise to improve lower limb muscle mass is conducive to the prevention of female osteoporosis.

## 1. Introduction

The aging population in China has been dramatically growing, which becomes a heavy burden for the government at all levels. In addition to the common metal diseases such as Alzheimer's disease and Parkinson's disease [1, 2], an increasing attention is paid to the physical diseases.

Osteopenia/osteoporosis (OP) is a metabolic bone disease mainly caused by aging, which is associated with gradual changes in body composition [3–6]. By means of the long-standing bone mass reduction and bone microstructure destruction, OP is making the appendicular bone brittler and brittler, which is prone to fracture. There are many known and potential driving factors influencing OP, for instance, the intake of vitamin D, hormone level, and sex-specific metabolic diseases [4]. Thus, the whole progression is entirely different between men and women [7, 8]. The population with abnormal bone mass in women is significantly higher than that in men [9], especially in postmenopausal women [4, 10]. As a hotspot, the association has been widely concerned between bone mineral density (BMD) and aging, body weight, nutritional status, smoking, alcohol, physical activity, etc. [11–13]. However, the research conclusions regarding the contribution to the adequate maintenance of BMD cannot reach a consensus [14–23]. Reid et al. took the lead in demonstrated that fat mass (FM), one main component of the body weight, is closely related to fat mass in premenopausal women [19]. Next year, the Framingham study stated that weight or BMI is much more strongly associated with BMD in elder women and men as a load factor [24]. Further, Dimitri et al. believed that obesity is a protective against fracture based on their study [25]. For postmenopausal women, Mpalaris and his colleagues proposed a U-bend curve to illustrate the relationship between BMI and the fracture risk [26]. For children, neither the diagnostic criteria is uniform nor the decision of therapy as well as therapeutic efficacy comes to reach agreement [8, 25, 27–32]. What is worse, the acataleptic relationship between body composition and BMD affects the diagnosis and treatments of the patients with other complex diseases [33–38].

The study conducted here is aimed at checking if different assemblies of body components may play different roles in bone metabolism. Should the further study on the correlation between body composition and bone health help to guide women to prevent and treat osteoporosis and improve their life quality?

## 2. Objects and Methods

### 2.1. Research Objects

Female employees of one university who had routine physical check-ups in the examination center of the Second Affiliated Hospital of Shandong First Medical University from January 2021 to May 2021 were initially recruited as the research objects. They had not participated in formal vocational physical exercise and voluntarily accepted DEXA monitoring bone mineral density and body composition analysis. Finally, 90 cases were included, aged 37-85 years, with an average of (54.84 ± 7.88) years. This study was approved by the ethics committee of the Second Affiliated Hospital of Shandong First Medical University, and all subjects signed informed consent. Specific inclusion criteria were as follows: (1) no disease affecting bone metabolism (thyroid disease, Xin syndrome, etc.); (2) no drugs affecting bone metabolism and body composition (glucocorticoid, estrogen, thyroid hormone, parathyroid hormone, calcitonin, diphosphate, etc.); (3) no serious liver and kidney diseases; (4) do not drink alcohol; and (5) no history of tumor.

### 2.2. General Data Collection

The subjects were fasting, took off their shoes, bareheaded, wearing single clothes, measured their weight (kg) and height (cm), and calculated their BMI. Calculation formula was as follows: weight (kg) divided by the square of height (m^2^). Based on the BMI grouping standard formulated by the working group on obesity in China (wgoc) and the guidelines in references [3, 5], the cohort with 18.5 ≤ BMI < 24 kg/m^2^ is the normal weight group, while the cohort with BMI ≥ 24 kg/m^2^ is the overweight/obese group.

### 2.3. Body Composition Test

Use the body 770 body composition tester to test the body composition of the subjects. The test indexes include waist hip ratio, muscle mass (kg), fat mass (kg), body fat percentage (%), upper limb muscle mass (kg), trunk muscle mass (kg), lower limb muscle mass (kg), upper limb fat mass (kg), trunk fat mass (kg), lower limb fat mass (kg), whole-body phase angle (°), and visceral fat area (cm^2^).

### 2.4. Bone Mineral Density Test

According to the Chinese expert consensus about the diagnosis of osteoporosis [39], the bone mineral density of lumbar spines 1-4 (L1-4) was tested by dual energy X-ray bone mineral density tester (Primus, OSTO, Korea) [40].

### 2.5. Statistical Analysis

The SPSS v22.0 statistical software is used for data analysis, and the measurement data are expressed by mean ± standard deviation (± s). The two samples were compared by *t*-test. Spearman was used to analyze the correlation between body composition and bone mineral density. The relationship between bone mineral density and body composition was analyzed by linear regression. The difference was statistically significant (*P* < 0.05).

## 3. Results

### 3.1. General Information

The screened 90 women were finally included in this study, age (54.84 ± 7.88) years, height (158.94 ± 5.30) cm, weight (65.37 ± 10.41) kg, and BMI (25.86 ± 3.87) kg/m^2^. The waist hip ratio and body fat percentage of the study group were higher than the normal level, and the body composition was (see Table 1 for details).

### 3.2. Comparison of Bone Mineral Density with Different BMI

According to the BMI grouping standard formulated by WGOC, the population is divided into the normal weight group and overweight/obesity group. By comparing the bone mineral density of lumbar spines L1-4 between the two groups, it can be seen that the bone mineral density of the overweight/obesity group is significantly higher than that of the normal weight group (see Table 2 for details).

### 3.3. Correlation Analysis and Multiple Regression Analysis between Body Composition and Bone Mineral Density

Spearman correlation analysis showed that age was negatively correlated with L1-4 BMD, and skeletal muscle, upper limb muscle, trunk muscle, lower limb muscle, and whole-body phase angle were negatively correlated with L1-4 BMD (see Table 3 for details).

### 3.4. Multiple Regression Analysis of Body Composition and Bone Mineral Density

Skeletal muscle, including upper limb muscle, trunk muscle, and lower limb muscle, was used as independent variables for multiple linear regression analysis. L1-4 bone mineral density is the dependent variable and age, and skeletal muscle and whole-body phase angle are the independent variables. Multiple linear regression analysis shows that age is the negative influencing factor of bone mineral density, and skeletal muscle is the protective factor of BMD (see Table 4 for details).

Taking L1-4 BMD as dependent variable and age, and upper limb muscle, trunk muscle, lower limb muscle, and whole-body phase angle as independent variables, linear regression analysis shows that age is a negative influencing factor of BMD, and lower limb muscle is a protective factor of BMD (see Table 5 for details).

## 4. Discussion

The outcomes of body composition analysis mainly provide the proportion of water, muscle, fat, and inorganic salts in the total body mass. These values can be used to evaluate the nutritional and energy metabolism status and overall health status of the body and can guide the diagnosis, treatment, and prognosis of a variety of diseases [41]. The present study suggests that lower limb muscle mass is a protective factor to keep the normal index of BMD in the female working in the city of Tai'an.

As early as the 1990s, the relationship between BMI, body weight, and bone health has been well studied, but the conclusions derived from different studies have not been consensual. Evans et al. illustrated that the areal BMD of the whole body, lumbar spine, hip, tibia, and radius of obese adults was higher than that with normal weight. Plus, the number of cortical bone and trabecular bone was significantly increased [17]. Yang and Shen also proved that the BMD of spine and femoral neck received a promotion accompanied with the increase of BMI and hip circumference [42]. However, Compston et al. reported an increased risk of ankle and femoral fractures in postmenopausal obese women [43]. The proportion of body compositions is various among the different populations, even they have the same body mass. The application of BMI or body weight alone cannot truly reflect the individual composition and health status of individuals.

In recent years, studies have shown that muscle mass and adipose tissue can affect bone mineral density. In our previous studies on male body composition and bone mineral density, we found that lean mass (LM) and lean body mass index (LBMI) play a decisive role in bone mineral density. In overweight/obese people, percentage body fat (% BF) and fat mass index (FMI) are negative factors of bone mineral density [44]. A study based on men over 50 years old shows that FMI is the protective factor of lumbar spine, and LBMI and fat free mass index (FFMI) are the protective factors of hip BMD [11]. Limb muscles are the protective factor of bone strength in female population, and subcutaneous adipose tissue is the risk factor of bone strength decline. This conclusion is not affected by menopause. The risk of osteoporosis increases with the decrease of total fat and lean tissue in postmenopausal women. Previous studies suggest that body composition plays different roles in bone health of different populations [10, 45]. In this study, there is no significant correlation between fat/obesity and bone mineral density in the female population. The effect of adipose tissue on bone health is still controversial and needs further research. Most studies have not seen further stratification analysis of whole-body muscles. However, it is found that there is a positive correlation between muscle and BMD [46]. Lower limb muscle mass is more conducive to the prevention of osteoporosis than body muscle and upper limb muscle. The possible protective mechanisms of muscle for bone health are as follows: (1) the gravity generated by muscle tissue through its own weight and the stress generated by muscle contraction on bone promote bone growth and development and increase BMD and bone strength. (2) Muscle produces insulin-like growth factor 1, fibroblast growth factor 21, myostatin, irisin, and other chemicals, which act on mesenchymal, osteoblasts, osteoclasts, and osteoblasts through paracrine to regulate bone metabolism [47, 48].

The limitation of this study is as follows: first of all, the sample size of objects is kind of small, which may lead to the bias in the results. Secondly, this study only detects the measurement of lumbar bone mineral density and cannot determine the correlation between bone mineral density and body composition in other parts. In future research, the sample size can be further expanded to further determine the reliability of the research results, and the monitoring parts of bone mineral density can be extended to femur bone mineral density of forearm and whole body to further verify the correlation between body composition and bone mineral density of various parts of the body.

There is a significant correlation between human body composition and bone health, but there are few studies with large sample on the correlation between bone health and human body composition in different populations. In clinic, we should pay more attention to the multiple measurements [42] and data analysis involving human body composition in the further studies, so as to improve the life quality of the patients.

## Figures and Tables

**Table 1:** General information about body composition of female employees.

Project	Minimum	Maximum	Mean (^−^*x*)	Standard deviation (*s*)
Age (y)	37	85	54.84	7.88
Height (cm)	146.1	171.3	158.94	5.3
Weight (kg)	46.5	101.8	65.37	10.41
BMI(kg/m^2^)	19.3	39.8	25.86	3.87
Waist hip ratio	0.83	1.11	0.94	0.061
Skeletal muscle mass (kg)	15.8	28.8	21.99	2.85
Body fat (kg)	13.2	51.9	24.68	7.4
Percentage of body fat (%)	25.6	52.7	37.15	6.05
Upper limb muscle mass (kg)	2.74	6.47	4.24	0.73
Trunk muscle mass (kg)	14.1	25.2	18.92	2.25
Lower limb muscle mass (kg)	8.37	15.97	12.34	1.77
Upper limb fat (kg)	1.6	11.3	3.75	1.66
Trunk fat (kg)	6.1	25.6	12.6	3.81
Lower limb fat (kg)	4	13.1	7.11	1.84
Visceral fat area (cm^2^)	54.4	262.6	127.68	43.83
Whole-body phase angle (°)	3.6	5.9	4.88	0.47
Lumbar 1-4 bone mineral density (g/cm^2^)	0.566	1.539	1.007	0.191

**Table 2:** Comparison of bone mineral density of different BMI.

BMI	*n*	Mean	Standard deviation	*t*	*P*
Normal weight group	33	0.943	0.207	-2.008	<0.05
Overweight group	37	1.039	0.195		

**Table 3:** Correlation analysis between body composition and bone mineral density.

Project	*r*	*P*
Age (y)	-0.43	<0.01
BMI (kg/m^2^)	0.251	<0.05
Waist hip ratio	-0.041	>0.05
Skeletal muscle mass (kg)	0.453	<0.01
Body fat (kg)	0.152	>0.05
Percentage of body fat (%)	0.059	>0.05
Upper limb muscle mass (kg)	0.388	<0.01
Trunk muscle mass (kg)	0.373	<0.01
Lower limb muscle mass (kg)	0.419	<0.01
Upper limb fat (kg)	0.138	>0.05
Trunk fat (kg)	0.144	>0.05
Lower limb fat (kg)	0.176	>0.05
Visceral fat area (cm^2^)	0.049	>0.05
Whole-body phase angle (°)	0.208	<0.05

**Table 4:** Linear regression analysis of body composition and bone mineral density.

Project	Standard *β* value	*P* value
Age (y)	-0.355	<0.01
Skeletal muscle mass (kg)	0.35	<0.01

**Table 5:** Linear regression analysis of body composition and bone mineral density.

Project	*r* value	*P* value
Age (y)	-0.333	<0.01
Lower limb muscle mass (kg)	0.618	<0.01

## Data Availability

No data were used to support this study.
